# The Efficacy and Safety of Xinjia Xuanbai Chengqi Granules in Acute Exacerbation of COPD: A Multicentre, Randomised, Double-Blind, Controlled Trial

**DOI:** 10.1155/2022/7366320

**Published:** 2022-06-23

**Authors:** Ruihan Qi, Hongchun Zhang, Demin Li, Feng Gao, Qing Miao, Sheng Chen, Yan Huang, Lei Wu, Zhenhui Lu, Haibo Hu, Erran Li, Zhibin Chen

**Affiliations:** ^1^Department of Respiratory and Critical Care Medicine, Shenzhen Hospital of Traditional Chinese Medicine, Shenzhen 518033, China; ^2^Center of Respiratory Medicine, China-Japan Friendship Hospital, Beijing 100029, China; ^3^Department of Respiratory Medicine, Wang Jing Hospital of CACMS, Beijing 100102, China; ^4^Department of Pulmonary Disease, Xiyuan Hospital of CACMS, Beijing 100091, China; ^5^Department of Pulmonary Disease, Inner Mongolia Autonomous Region Hospital of Traditional Chinese Medicine, Hohhot 750306, China; ^6^Department of Respiratory Medicine II, Hebei Hospital of Traditional Chinese Medicine, Shijiazhuang 050011, China; ^7^Respiratory Research Institute of Longhua Hospital, Shanghai University of Traditional Chinese Medicine, Shanghai 200032, China; ^8^Department of Respiratory and Critical Care Medicine, Qingdao Haici Medical Group, Qingdao 266033, China; ^9^Department of Respiratory and Critical Care Medicine, The First Hospital of China Medical University, Shenyang 110002, China; ^10^Department of Respiratory Medicine, The Second Affiliated Hospital of Fujian University of Traditional Chinese Medicine, Fuzhou 350002, China

## Abstract

**Purpose:**

The study aimed to explore the efficacy and safety of Xinjia Xuanbai Chengqi granules (XJXBCQ) combined with conventional medicine in the treatment of acute exacerbation of chronic pulmonary disease (AECOPD). *Patients and Methods*. This multicentre, double-blind, parallel, placebo-controlled, randomised clinical trial conducted in China from January 2019 to February 2021 recruited 330 participants who were allocated into three groups. All participants underwent conventional basic treatment with oxygen therapy, antibiotics, and a bronchodilator. Besides, group *A* received XJXBCQ granules and budesonide suspension for inhalation; group *B* received XJXBCQ granules and half dosage of budesonide suspension; and group *C* received budesonide suspension and a placebo. All therapies lasted for 5 days, and participants were followed up for 30 days after discharge. The primary outcomes were efficacy, traditional Chinese medicine (TCM) syndrome score, and clinical symptom score. Secondary outcomes included the blood gas analysis, serum inflammatory markers, adverse events, mortality, theoretical discharge time, actual hospitalisation time, proportion of patients requiring invasive mechanical ventilation, proportion of patients transferred to an intensive care unit (ICU), and readmission rate within 30 days after discharge.

**Results:**

XJXBCQ adjunct with conventional treatment could significantly improve the total efficacy (*P* < 0.05). Meanwhile, group *A* showed significantly better results than group *C* in the TCM syndrome score, phlegm score, and Wexner constipation score (*P* < 0.05). For modified British medical research council (mMRC), on day 3 (−0.17, 95% confidence interval [CI]: −0.33–−0.01) and day 4 (−0.20, 95% CI: −0.39–−0.02), group *A* performed statistically better than group *C*. No significant differences in other secondary outcomes were detected.

**Conclusion:**

XJXBCQ is beneficial and safe for AECOPD treatment and could be considered an adjunctive therapy for promoting the relief of clinical symptoms. This trial is registered with ChiCTR1800016915.

## 1. Introduction

Chronic obstructive pulmonary disease (COPD), characterised by persistent respiratory symptoms and airflow limitation, has become the fourth leading cause of death worldwide [1–3]. About 1 million COPD patients die in China every year, accounting for 31.1% of the total COPD deaths in the world [4]. The current incidence of COPD in China has risen from 8.2% to 8.6%, and the incidence in people over 40 years is 13.7%, increasing by about 67% compared with 2002 [5]. Given that COPD can be prevented, effective prevention and treatment will help diminish the acute exacerbation and postpone the disease progression. COPD management is still fundamentally heavily dependent on the use of bronchodilators and corticosteroids. Since long-term use of corticosteroids can result in adverse effects, and inflammation in COPD lungs is often poorly responsive to corticosteroid treatment, bronchodilators can hardly reverse the airflow obstruction. There is an urgent need for an alternative, more effective, and safer therapeutic approach that will not only relieve symptoms but also influence the natural course of COPD by preventing disease progression or even have the ability to reverse the disease [6, 7].

Complementary treatment, whose efficacy was confirmed by many studies, has been widely used in many chronic diseases as an alternative therapy to conventional medicines [8–11]. Traditional Chinese medicine (TCM), characterised by the theory of syndrome differentiation and overall conditioning, implies its potential advantages in the treatment of COPD. A systematic review has revealed that TCM combined with conventional medicines could accelerate the relief of clinical symptoms in COPD patients and improve lung function, modified British medical research council (mMRC), COPD assessment test (CAT), Saint George's respiratory questionnaire (SGRQ), 6-minute walking distance (6MWD), BMI, obstruction, dyspnoea, exercise capacity (BODE) score, and COPD patient-reported outcomes (COPD-PRO) to improve the quality of life and reduce the frequency of acute exacerbations and hospitalisation duration of AECOPD patients [12, 13]. Moreover, studies on TCM syndrome have found that in addition to respiratory symptoms, such as cough, phlegm, and wheezing, patients in acute exacerbation often experience constipation, abdominal distension, and yellow greasy tongue coating. Based on TCM theory, stating that the “lung and the large intestine are interior-exterior,” physicians offering the therapeutic approach called Tongfu Xiere, meaning treating both lung and gut, usually achieve good clinical outcomes in AECOPD treatment, and Xinjia Xuanbai Chengqi granules (XJXBCQ) is the representative formula of this kind of therapy. We implemented this rigorously designed clinical trial with the aim of validating the efficacy and safety of XJXBCQ in the treatment of AECOPD and understanding whether TCM therapy works better than conventional treatment.

## 2. Patients and Methods

### 2.1. Design

This was a multicentre, double-blind, randomised, placebo-controlled clinical trial conducted in China from October 2018 to March 2020 expectedly, aiming to recruit 360 participants from the respiratory inpatients. In this study, the block randomisation method was adopted, and participants with random numbers, 001–360, were randomly divided into three groups at a ratio of 1 : 1 : 1. The allocated medications of integrated Chinese and Western medicine for group *A* (group *A*), integrated Chinese and Western medicine for group *B* (group *B*), and Western standard medicine for group *C* (group *C*) were exactly the same in appearance, packaging, and specifications and were coded by professionals not participating in the statistical analysis of this project. The trial was registered at the Chinese Clinical Trial Registry (trial registration number: ChiCTR1800016915). Further information could be found in the published study protocol [14].

### 2.2. Ethics and Consent

Before randomisation, participants were asked to sign informed consent. The study was approved by the leading research unit, the Ethical Committee of China-Japan Friendship Hospital (ethics approval number: 2018-58-K40-4) and another ethical committee of research units participating in the study.

### 2.3. Inclusion and Exclusion Criteria

As the study protocol reported [14], AECOPD patients of clinical-grade severity of I–II [1, 15] with a syndrome of heat-phlegm and sthenic-fu, in the age range from 40 to 80 years, who volunteered to participate in the study and signed the informed consent were included in this trial. Meanwhile, patients who met any of the following criteria were excluded: (1) patients complicated with asthma, pneumonia, bronchiectasis, cystic fibrosis, pulmonary tuberculosis, lung cancer, or any other airflow-limiting disease with known causes and characteristic pathology; (2) patients complicated with coronary heart disease, hypertensive heart disease, or heart valve disease; (3) patients needing invasive mechanical ventilation; (4) patients with clinically confirmed or highly suspected pulmonary embolism; (5) patients with severe diseases of cardiovascular, cerebrovascular, hepatorenal, haematopoietic, or endocrine system; (6) patients with intestinal obstruction requiring surgical intervention; (7) pregnant or lactating patients; (8) mentally handicapped patients; (9) patients with alanine aminotransferase (ALT) and aspartate aminotransferase (AST) >1.5 times the upper limit of normal reference or serum creatinine (Scr) above the upper limit of normal reference; (10) patients requiring immunosuppressants; (11) patients taking oral or intravenous antibiotics before screening for more than 3 days in the last 3 months; (12) patients allergic to the basic therapeutic drugs, Chinese herbal medicinal ingredient prescription, or other substances prescribed through the research; (14) patients who have participated in or are participating in other clinical trials in the last 3 months; and (15) patients who were considered inappropriate to participate in this clinical trial by the investigator.

### 2.4. Intervention and Comparator

According to the protocol [14], all participants underwent conventional basic treatment with oxygen therapy, antibiotics (0.5 g levofloxacin hydrochloride intravenous injection once a day), and bronchodilator (500 ug ipratropium bromide solution for inhalation three times a day). Besides, group *A* received XJXBCQ granules (5 g, three times a day) and budesonide suspension for inhalation (2 mg Pulmicort Respules two times a day); group *B* received XJXBCQ granules (5 g, three times a day) and budesonide suspension for inhalation (1 mg Pulmicort Respules two times a day); and group *C* received the placebo of XJXBCQ granules (5 g, three times a day) and budesonide suspension for inhalation (2 mg Pulmicort Respules two times a day). All therapies lasted for 5 days. XJXBCQ (2.5 g/bag, batch number: 180605) and the related placebo were produced and packaged by Anhui Jiren Pharmaceutical with the China Pharmaceutical Production License (number: Wan 20160083). The details of the components of XJXBCQ are shown in Table 1 [14].

### 2.5. Measures

As previously reported [14], the primary outcomes were total efficacy (clinical recovery rate, markedly effective rate, and effective rate, explained in the protocol); clinical symptom scores including cough, 24 h phlegm, Wexner constipation score, and mMRC; and TCM syndrome score. The TCM syndrome score consisted of five symptoms: cough, dyspnoea, abdominal distension, constipation, and fever, and the evaluation criteria are available in the protocol [14]. These outcomes would be measured at baseline (day 1 [D1] to day 5 [D5] during the intervention) and day 6 (D6)—the first day after intervention. The evaluation criteria were explained in detail in the protocol [14]. The secondary outcomes were blood gas analysis (pH, PaO_2_, and PaCO_2_), recorded at baseline and day 6, and serum inflammatory markers (procalcitonin [PCT], C-reactive protein [CRP], interleukin [IL]-6, and tumour necrosis factor [TNF]-*α*) detected on baseline D3 and on D6. The safety outcomes of blood and urine routine; liver function (AST, ALT, total bilirubin [TBil], alkaline phosphatase [ALP], gamma-glutamyl transferase [GGT]), kidney function (blood urea nitrogen [BUN], estimated glomerular filtration rate [eGFR]); and electrocardiogram (ECG) were assessed at baseline and day 6. The adverse events were recorded at any time if they occurred. Other outcomes included mortality, theoretical discharge time, actual hospitalisation time, proportion of patients requiring invasive mechanical ventilation, proportion of patients transferred to an ICU, and readmission rate within 30 days after discharge.

### 2.6. Administration

As the leading unit of the research, China-Japan Friendship Hospital offered the standard operating procedures (SOPs) for all participating units. Researchers involved underwent a series of training sessions to guarantee a thorough understanding of research protocol and SOPs and ensure the accuracy of recorded data. The clinical data were first recorded in case report form (CRF) and then were electronically dually input into the Electronic Data Capture system. The Beijing Qihuang Pharmaceutical Clinical Research Center was employed as an independent quality inspector for monitoring and managing this trial.

### 2.7. Statistical Analysis

Statistical analysis was performed by SAS V. 9.4 software. For continuous variables, the paired *t*-test was used to compare the changes in clinical symptom scores before and after intervention, and the covariance analysis model was used for comparison between the groups. The multiplier method was used to calculate the quartiles (25%, 50%, and 75%) of time from enrolment to events occurring, and a bilateral 95% confidence interval (CI) and the incidence rate at each time point after enrolment were calculated. Kaplan–Meier curves were plotted using the log-rank test to compare theoretical hospital stay and actual hospital stay. For the binary variables, such as the recurrence rate of laboratory indicators, the all-cause mortality, the proportion of mechanical ventilation, the proportion of patients transferred to an ICU, and the proportion of readmission within 30 days after discharge, the 95% CI was calculated using a centrally stratified Cochran–Mantel–Haenszel *χ*^2^ test according to the classification, indicators, time points, quantity, and percentage.

## 3. Results

### 3.1. Sample Characteristics

The study was conducted between January 2019 and February 2021 in China. The trial had planned to recruit 360 participants, but eventually, a total of 331 eligible patients were screened, and 330 patients were actually enrolled, with 110 patients in group *A*, 109 patients in group *B*, and 111 patients in group *C*. Twenty-two patients failed to complete the trial, and the dropout rate was 5.45% in group *A*, 8.26% in group *B*, and 6.31% in group *C*. Participants accepting at least one time of treatment were included in the full-analysis set (FAS) and safety analysis set (SS), and those who completed all the treatment according to the protocol were admitted in per-protocol set (PPS). The patient enrolment distribution diagram is presented in Figure 1. As shown in Table 2, gender, age, vital signs, past history, and allergic history of allocated participants showed no statistical difference (*P* < 0.05). The three groups were also comparable in terms of acute exacerbation (AE) times within the last year, hospitalisation times for AE, FEV_1_%, and efficacy outcomes (*P* > 0.05).

### 3.2. Primary Outcomes

#### 3.2.1. Efficacy

The total efficacy rate was 90.75% in group *A* (9 clinical recovery, 31 markedly effective, 56 effective, and 10 invalid), 82.24% in group *B* (9 clinical recovery, 27 markedly effective, 52 effective, and 19 invalid), and 71.82% in group *C* (5 clinical recovery, 22 markedly effective, 52 effective, and 31 invalid), showing significant statistical difference between the three groups (*P*=0.0038). Besides, compared with group *C*, the total efficacy rate of group *A* was significantly better (*P* < 0.05). However, there was no statistical difference between group *A* and group *B* (Table 3).

#### 3.2.2. TCM Syndrome Score and Clinical Symptom Score

After a 5-days intervention, the TCM syndrome score and clinical symptom score (phlegm, mMRC, and Wexner score) were significantly improved in all three groups; meanwhile, group A performed significantly better than group C in TCM syndrome score, phlegm score, and Wexner constipation score (*P* < 0.05). For mMRC, there was no statistical difference between the three groups on D6, but on the third and fourth days of the intervention (D3, D4), group *A* performed statistically better than group *C* (D3: −0.17, 95% CI: −0.33–−0.01; D4: −0.20, 95% CI: −0.39–−0.02). Based on conventional Western medicines, adjunctive traditional Chinese medicine was more adept in relieving clinical symptoms of AECOPD patients (Table 3).

### 3.3. Secondary Outcomes

#### 3.3.1. Blood Gas Analysis and Serum Inflammatory Markers

For blood gas analysis measured on day 6 compared with baseline, only group *A* showed improved PaO_2_. No statistical difference was shown after intervention for pH and PaCO_2_ between the three groups (Table 3). Regarding serum inflammatory markers (CRP, IL6, PCT, and TNF-*α*), only a few patients showed abnormal values at baseline, although the level of inflammatory factors seemed to be lower on D6 after the intervention; however, there were no statistical differences between D6 and baseline (Table 3). Moreover, we used the recovery rate of serum inflammatory markers on D6 to represent the anti-inflammatory effect of the three treatments; however, no difference was observed after intervention or between the three groups (Table 4).

### 3.4. Adverse Events

Fifteen participants (2 from group *A*, 8 from group *B*, and 5 from group *C*) reported 20 adverse events (4.57%), which were relevant to the given intervention judged by researchers. The most frequent adverse event was diarrhoea, and other event types are listed in Table 5. There were two serious adverse events: a patient in group *A* suspended the trial for severe diarrhoea and vomit that resolved after quitting the drug, and another patient in group *C* suffered drug-induced hypersensitivity, considered to be a severe adverse event by researchers. Other adverse events were mild to moderate (Table 5).

### 3.5. Other Outcomes

The median length of hospitalisation of the three groups was 8 days, 9 days, and 8 days, respectively, showing no statistical difference (*P*=0.6635). Two patients (1.89%) in group *A* and two patients in group *B* (1.87%) were readmitted due to AECOPD within 30 days after discharge, and the readmission rate of the three groups was similar (*P*=0.3624). A patient died in group *A* due to acute cerebral infarction that did not relate to the study intervention. Another patient in group *C* was transferred to an ICU during hospitalisation for requiring invasive mechanical ventilation. Mortality, proportion of patients requiring invasive mechanical ventilation during hospitalisation, and proportion of patients transferred to an ICU during hospitalisation of the three groups showed no statistical difference (*P*=0.3614; *P*=0.3711; *P*=0.3711).

### 3.6. Discussion

Patients with chronic respiratory disease are two to three times more likely to have gastrointestinal issues, and COPD patients have had higher incidences of inflammatory bowel disease (IBD) compared to non-COPD controls, while over a half of IBD patients, in contrast, show pulmonary involvement [9, 10]. Of COPD patients, 40% have had irregular stools compared to 15% of non-COPD patients when hospitalised, showing statistical difference [16]. Moreover, constipation has been positively correlated with the severity of dyspnoea, acute exacerbation times, and complication of COPD [17]. As for clinical symptoms, these peripheral disease manifestations highlight the immunological crosstalk between the lung and gut, the two mucosal sites, termed the gut-lung axis, whereby the immunological health of the gut impacts the health of the lung [18], similar to the TCM theory arguing that “the lung and the large intestine are interior-exterior,” which postulates that the disruption of interactive networks (Biao-Li) between these two related organ systems may disrupt the bidirectional gut-lung communication, leading to the onset of a disease. Thus, it has been a common strategy for TCM practitioners to simultaneously treat the lung and gut in respiratory diseases, including AECOPD, which is often accompanied by constipation and abdominal distension. Moreover, XJXBCQ is a representative formula of the gut-lung correlation theory.

The results of this study demonstrated that XJXBCQ significantly reduced clinical symptoms of AECOPD patients compared with conventional medicine. Judging from the Guidelines for TCM Diagnosis and Treatment of COPD (2011) [19] and Guidelines for Clinical Research of New TCM for Chronic Bronchitis (2002) [20], the total TCM syndrome score and the efficacy rate of combination therapy of XJXBCQ and conventional medicine were superior to using conventional medicine alone, especially in relieving dyspnoea, phlegm, abdominal distension, and constipation. Additionally, the mMRC, the Wexner constipation score, and the 24-hour phlegm score also showed improvement after the combination therapy. However, there were no differences in the recovery rate of IL6, CRP, PCT, and TNF-a, possibly due to the mild degree of inflammation for most AECOPD participants whose inflammatory markers were normal when allocated.

For blood gas analysis, PaO_2_ was significantly improved after the intervention involving combination therapy. Although there were no statistical differences, PaCO_2_ values were slightly elevated in the three groups. We assumed that the diaphragm mobility was limited to some extent as all enrolled patients had a certain degree of abdominal distension and constipation. Once abdominal distension and constipation were relived after the intervention, the diaphragm mobility might have improved, dyspnoea improved, respiratory rates slowed down, and CO_2_ emission decreased, leading to an increase in PaCO_2_ as a consequence.

In this trial, we set three groups to understand whether the combination of XJXBCQ with conventional medicine could reduce the use of corticosteroids as many COPD patients show poor response to the anti-inflammatory benefits of corticosteroids, and the use of inhaled corticosteroids (ICSs) has been associated with an increased risk of pneumonia in patients with COPD [7, 21]. However, although no statistical difference was found in the comparison between group *A* and group *B* for detected outcomes, it should be prudent to reduce corticosteroids while using XJXBCQ due to the lack of rigorous evidence.

Regarding safety, the incidence of drug-related adverse events was similar in the three groups, and the recorded events mainly involved gastrointestinal disorders, including diarrhoea and vomiting. Given that XJXBCQ itself has a laxative effect, which may cause diarrhoea, prudent judgement should be taken regarding whether diarrhoea could be regarded as an adverse reaction.

This multicentre, double-blind, randomised trial was conducted strictly according to the protocol, showing clinical benefits of XJXBCQ in treating AECOPD. Nevertheless, several limitations still exist. We aimed to recruit AECOPD patients with clinical-grade severity of I–II, but actually, most of the patients allocated were mild to moderate and at grade I severity; consequently, many outcomes, such as the blood gas analysis and serum inflammation markers, were normal at baseline, which makes it impossible to assess the effect of the intervention on them, as well as the outcomes of mortality, the proportion of patients requiring invasive mechanical ventilation during hospitalisation, and the proportion of patients transferred to an ICU during hospitalisation.

## 4. Conclusions

The results of this study demonstrated that the use of XJXBCQ in AECOPD adjunctively with conventional medicine for 5 days could significantly accelerate the recovery of clinical symptoms of dyspnoea and phlegm, the mMRC score, and the specific symptoms of abdominal distension and constipation, as well as improving PaO_2_, indicating that XJXBCQ simultaneously treating the lung and gut was effective and safe. Moreover, the results also corroborate the importance of the gut-lung axis in AECOPD treatment. Further basic research is needed to explore the mechanism by which XJXBCQ relieves AECOPD through the gut-lung axis.

## Figures and Tables

**Figure 1:** A diagram of the study flow.

**Table 1:** Main components of Xinjia Xuanbai Chengqi granules.

Chinese name	English common name	Scientific name	Amount (grams)
Ku Xing Ren	Bitter almonds	*Armeniacae Semen Amarum*	6
Sheng Shi Gao	Gypsum	*Gypsum Fibrosum*	15
Gua Lou	Snakegourd fruit	*Trichosanthis Fructus*	9
Da Huang	Rhubarb	*Rhei Radix et Rhizoma*	6
Huang Qin	Baikal skullcap root	*Scutellariae Radix*	9
Zi Su Zi	Perilla fruit	*Perillae Fructus*	9
Zhi Gan Cao	Licorice root	*Glycyrrhizae Radix et Rhizoma Praeparata Cum Melle*	6
Jin Qiao Mai	Wild buckwheat rhizome	*Fagopyri Dibotryis Rhizoma*	10
Zi Wan	Tatarian aster root	*Asteris Radix et Rhizoma*	9

**Table 2:** Demographic characteristics and baseline data of the participants.

Item	Group A (*n* = 106)	Group B (*n* = 107)	Group C (*n* = 110)	Statistics	*P* value
Gender					
Male	75	86	92	5.86	0.053
Female	31	21	18		
Age (years)	67.17 ± 8.06	68.45 ± 7.28	68.28 ± 8.42	0.82	0.442
Vital signs					
Temperature (°C)	36.52 ± 0.51	36.46 ± 0.37	36.44 ± 0.43	0.91	0.402
Heart rate (times/min)	85.32 ± 13.20	82.70 ± 11.73	84.79 ± 11.34	1.40	0.248
Respiratory rate (times/min)	20.36 ± 1.74	20.31 ± 1.80	20.17 ± 2.18	0.27	0.762
SBP (mmHg)	134.34 ± 17.40	132.09 ± 18.46	133.01 ± 17.32	0.43	0.650
DBP (mmHg)	80.12 ± 9.44	78.51 ± 10.34	78.82 ± 10.97	0.73	0.481
Past history (%)	91 (85.85)	94 (87.85)	97 (88.18)	0.32	0.853
Allergic history (%)	21 (19.81)	26 (24.30)	27 (24.55)	0.89	0.640
AE times within last year	1.18 ± 1.01	1.17 ± 1.33	1.08 ± 1.17	0.22	0.804
Hospitalisation times for AE	0.80 ± 0.83	0.81 ± 0.80	0.78 ± 1.04	0.04	0.962
FEV_1_% (numbers)	52.35 ± 14.84 (62)	51.19 ± 14.75 (63)	52.32 ± 13.27 (67)	0.14	0.872
Efficacy outcomes					
Phlegm score	38.08 ± 25.19	41.30 ± 29.78	38.53 ± 50.05	0.24	0.786
Wexner score	7.17 ± 3.56	7.55 ± 3.71	7.05 ± 3.64	0.55	0.577
mMRC	2.35 ± 0.81	2.38 ± 0.75	2.25 ± 0.84	0.76	0.470
pH	7.41 ± 0.03	7.40 ± 0.04	7.40 ± 0.04	0.61	0.545
PaO_2_ (mmHg)	75.49 ± 20.79	76.30 ± 21.07	77.19 ± 30.49	0.12	0.886
PaCO_2_ (mmHg)	41.55 ± 9.44	42.73 ± 9.92	42.54 ± 14.35	0.30	0.741
TCM syndrome score	5.58 ± 2.21	5.47 ± 2.25	5.29 ± 2.15	0.46	0.631

Note. SBP: systolic blood pressure; DBP: diastolic blood pressure; AE: acute exacerbation; TCM: traditional Chinese medicine; mMRC: modified British medical research council.

**Table 3:** Comparison of outcomes after intervention.

Variable	Group	$\bar{X}\pm s$		D6–baseline	
		Baseline	D6	$\bar{X}\pm s$	*P* value
TCM syndrome score	Group *A* (*n* = 106)	23.32 ± 6.74	9.11 ± 6.18^*∗*^^#^	−14.21 ± 7.29	<0.0001
	Group *B* (*n* = 107)	22.99 ± 7.44	9.84 ± 6.30	−13.15 ± 7.42	<0.0001
	Group *C* (*n* = 110)	22.53 ± 6.34	11.54 ± 6.52	−10.99 ± 8.36	<0.0001

Phlegm	Group *A* (*n* = 106)	1.63 ± 0.81	0.64 ± 0.57^*∗*^	−0.99 ± 0.81	<0.0001
	Group *B* (*n* = 107)	1.68 ± 0.73	0.71 ± 0.61	−0.97 ± 0.81	<0.0001
	Group *C* (*n* = 110)	1.57 ± 0.80	0.86 ± 0.77	−0.71 ± 1.09	<0.0001

mMRC	Group *A* (*n* = 106)	2.35 ± 0.81	1.42 ± 0.99	−0.93 ± 0.89	<0.0001
	Group *B* (*n* = 107)	2.38 ± 0.75	1.50 ± 0.83	−0.88 ± 0.75	<0.0001
	Group *C* (*n* = 110)	2.25 ± 0.84	1.56 ± 0.90	−0.69 ± 0.89	<0.0001

Wexner	Group *A* (*n* = 106)	7.17 ± 3.56	3.25 ± 2.71^*∗*^	−3.92 ± 2.69	<0.0001
	Group *B* (*n* = 107)	7.55 ± 3.71	3.75 ± 3.00	−3.80 ± 3.28	<0.0001
	Group *C* (*n* = 110)	7.05 ± 3.64	4.11 ± 3.48	−2.95 ± 3.03	<0.0001

pH	Group *A* (*n* = 100)	7.41 ± 0.03	7.40 ± 0.03	−0.00 ± 0.03	0.1212
	Group *B* (*n* = 96)	7.40 ± 0.04	7.40 ± 0.04	−0.00 ± 0.03	0.4060
	Group *C* (*n* = 104)	7.40 ± 0.04	7.40 ± 0.04	−0.00 ± 0.03	0.5197

PaO_2_	Group *A* (*n* = 100)	75.49 ± 20.79	80.81 ± 23.28	4.49 ± 18.39	0.0165^*∗*^
	Group *B* (*n* = 96)	76.30 ± 21.07	78.63 ± 26.01	1.87 ± 26.44	0.4896
	Group *C* (*n* = 104)	77.19 ± 30.49	78.53 ± 23.72	0.91 ± 31.60	0.7703

PaCO_2_	Group *A* (*n* = 100)	41.55 ± 9.44	42.25 ± 9.10	0.68 ± 4.70	0.1488
	Group *B* (*n* = 96)	42.73 ± 9.92	43.65 ± 12.62	1.10 ± 7.10	0.1313
	Group *C* (*n* = 104)	42.54 ± 14.35	43.45 ± 14.11	1.00 ± 5.36	0.0596

CRP	Group *A* (*n* = 101)	11.98 ± 29.33	8.27 ± 23.02	−3.61 ± 17.50	0.0408
	Group *B* (*n* = 102)	16.12 ± 33.67	9.35 ± 30.50	−6.60 ± 28.62	0.0218
	Group *C* (*n* = 103)	15.60 ± 35.21	8.13 ± 23.61	−7.44 ± 24.03	0.0022

PCT	Group *A* (*n* = 102)	0.09 ± 0.16	0.08 ± 0.15	−0.02 ± 0.28	0.4015
	Group *B* (*n* = 100)	0.09 ± 0.11	0.08 ± 0.10	−0.02 ± 0.12	0.0926
	Group *C* (*n* = 103)	0.06 ± 0.06	0.07 ± 0.06	−0.00 ± 0.06	0.4863

IL6	Group *A* (*n* = 93)	12.35 ± 21.63	11.02 ± 13.91	−0.77 ± 17.53	0.6730
	Group *B* (*n* = 94)	11.58 ± 17.60	25.41 ± 139.20	15.01 ± 142.62	0.3103
	Group *C* (*n* = 98)	21.84 ± 101.39	10.14 ± 14.05	−12.72 ± 101.52	0.2177

TNF-*α*	Group *A* (*n* = 91)	14.37 ± 29.37	14.04 ± 29.01	−0.30 ± 24.16	0.9044
	Group *B* (*n* = 92)	72.41 ± 235.71	59.68 ± 210.30	−10.49 ± 209.31	0.6319
	Group *C* (*n* = 100)	49.39 ± 181.27	32.40 ± 139.82	−15.91 ± 177.03	0.3711

Note. ^*∗*^*P* < 0.05, group *A* compared with group *C*; ^#^*P* < 0.05. D6: the day after intervention; TCM: traditional Chinese medicine; mMRC: modified British medical research council.

**Table 4:** The recovery rate of serum inflammatory markers.

Groups	CRP			PCT			IL6			TNF-*α*		
	*n*	*n* ^*∗*^	Rate (%)	*n*	*n* ^*∗*^	Rate (%)	*n*	*n* ^*∗*^	Rate (%)	*n*	*n* ^*∗*^	Rate (%)
Group *A*	25	12	48.00	12	2	16.67	15	4	26.67	13	3	23.08
Group *B*	30	13	43.33	18	5	27.78	22	8	36.36	11	2	18.18
Group *C*	31	17	54.84	8	2	25.00	16	8	50.00	15	2	13.33
*P* value	0.6373			0.5082			0.4462			0.8747		

Note. *n*: numbers of participants with abnormal inflammatory markers at baseline; *n*^*∗*^: numbers of participants having abnormal inflammatory markers and returning to normal on the day after intervention (day 6). CRP: C-reactive protein; PCT: procalcitonin; IL6: interleukin-6; TNF-*α*: tumour necrosis factor-*α*.

**Table 5:** Summary of adverse events.

Event type	Group *A* (no. of cases)	Group *B* (no. of cases)	Group *C* (no. of cases)
Diarrhoea	1	2	1
Vomit	1	1	0
High blood pressure	1	2	0
Insomnia	0	2	0
Dizziness	0	2	1
Dyspnoea	0	3	0
Itchy skin	0	0	1
Stomach upset	0	0	1
Drug-induced hypersensitivity	0	0	1

## Data Availability

The metadata of the trial were uploaded to National Population Health Data Center of China (https://www.ncmi.cn/phda/projectDataDetail.html?id=93e9e1aa-4444-3f78-9d30-17f7bbf93ad7), and it will be accessible from 30 June, 2024.
